RETRACTED

# Analysis on the Characteristics and Influence of the Teaching Environment Design of College Politics Course under the Campus Humanistic Governance Environment

**DOI:** 10.1155/2022/1703167

**Published:** 2022-08-10

**Authors:** Jian Gao, Bo Li

**Affiliations:** Sichuan Water Conservancy College, Chengdu 611231, China

## Abstract

This paper discusses the characteristics and influence of the teaching environment design of College Politics Course under the campus humanistic governance environment. Based on Rogers' humanistic theory in the campus humanistic governance environment, this paper designs the teaching environment of college politics course from the aspects of learning situation analysis, teaching method design, teaching content design, teaching objectives and process design, and teaching evaluation design. Through the way of scoring, we evaluate the impact of environmental design on teaching. *Results*. After the design of teaching environment, the scores of teachers were (8.21 ± 1.22), (7.84 ± 1.20), (9.25 ± 0.12), and (9.10 ± 0.51), respectively, in terms of vivid and intuitive teaching methods and means, method innovation, teacher-student interaction, and knowledge expansion. Students' scores were (8.65 ± 4.10), (8.52 ± 1.00), (9.33 ± 0.16), and (8.77 ± 0.54), respectively, and other teaching conditions were also improved. *Conclusion*. Based on the campus humanistic governance environment, designing the teaching environment of college politics course can effectively improve the teaching effect and teaching quality.

## 1. Introduction

In the 21st century, we are in an era of rapid development of information. Social progress has brought changes in life needs. People begin to pay attention to the realization of self-worth and seek a stage to show themselves. As an important part of the society, the classroom is their stage, which requires classroom teaching to pay attention to students' own development, give more students the opportunity to show their abilities, and meet their emotional needs [1]. Teaching design (Figure 1) is also the premise of classroom teaching. How to make teaching design adapt to students' development, mobilize students' emotions, and realize students' potential is a problem in front of teachers.

Ideological and political subject is a course with its special nature, which is reflected in its moral education. Therefore, the teaching design of the ideological and political course should reflect the student-centered, grasp the students' moral feelings, carry out knowledge education, and realize the combination of knowing and making the students' personality perfect and developed. This design is also in line with the requirements of the new curriculum reform for teaching to promote students' all-round development, meet students' needs, and cultivate learning ability. However, the authors found that these requirements have not been well implemented in the ideological and political teaching design in colleges and universities, and there are problems such as teachers' filling the hall and ignoring students' participation. The reason may be that teachers lack the theoretical guidance related to humanism and the reference of teaching design mode [2, 3]. Rogers' humanistic theory puts forward the concepts of meaningful free learning and informed unity and believes that learning is a process of students' autonomy and self-consciousness. He relies on teachers to guide the combination of learning content and students' personal meaning to achieve the common development of cognition and emotion, and teaching should achieve the realization of students' integrity. Therefore, the author believes that Rogers' humanistic theory (Figure 2) is adapted to the needs of contemporary people's development and the teaching concept of Ideological and political discipline. According to Rogers' humanistic theory, the design of teaching design with students as the main body and emotion as the main line is of great significance to ensure and improve the quality of Ideological and political teaching.

RETRACTED

## 2. Literature Review

The three-generation teaching design is divided into two directions as a whole. The first direction is “teaching,” and the second direction is “learning.” “Teaching” mainly focuses on the first- and second-generation teaching design, mainly studying what teachers teach and how to teach and paying less attention to students' learning problems. In terms of behaviorism, Thorndike put forward the “theory of trial and error” and believed that teaching should be a combination of preparation, connection, and effect evaluation. According to his theory, he set up a set of teaching design models about the teaching process [4]. Skinner's operational learning theory holds that the essence of learning is to reflect the change of probability, and reinforcement is a tool to enhance the reflection of probability. It further proposes that the teaching design should pay attention to the students' own status, give them the right to set their own pace, and actively give reinforcement and feedback. In terms of cognitivism (Figure 3). Gagne's information processing learning theory is particularly significant to teaching design. Gagne believes that learning is a process of information processing, and this internal information processing process is closely related to external teaching events. Gagne divides teaching into eight stages, and the design of teaching process should reflect these eight stages and should be sequential [5].

RETRACTED

“Learning” is mainly represented by constructivism and humanism, highlighting the status of students in the teaching process and focusing on how to help students improve their learning efficiency and realize their self-worth. Constructivism believes that education should “grow” new knowledge with students' original knowledge and experience, and it has developed teaching methods such as immediate access teaching, scaffolding teaching, and anchor teaching, which enrich the theory of teaching design. In terms of humanism, Rogers put forward “meaningful free learning,” which emphasizes the relationship between learning content and individuals, highlights the unity of knowledge, requires learners to choose learning materials on their own within a considerable range, arranges learning scenarios suitable for themselves, and expands new connotations for teaching design [6, 7].

In 2004, the release of “Ideological and Political Curriculum Standard (Experiment)” in Colleges and universities brought a new upsurge of ideological and political teaching design research. The author has found three books related to teaching design through a library, mainly including Hutiangeng's “middle school ideological and political teaching design and case study,” Kuang Lizhan's “ideological and political subject teaching design,” and Liuwenchuan's “new ideological and political course teaching design and evaluation in Colleges and universities.” Among them, “middle school ideological and political teaching design and case study” analyzes various elements of ideological and political teaching design in detail and attaches actual teaching cases to build a theoretical framework and operation mode of teaching design with discipline characteristics. “Ideological and political subject teaching design” studies the related problems in ideological and political teaching design, absorbs the excellent achievements of existing teaching design, expands the conceptual foundation, and gives help to ideological and political teaching design at the theoretical level. Based on 30 real cases, the “teaching design and evaluation of the new ideological and political course in colleges and universities” makes a real analysis of the teaching content, students' learning situation (Figure 4), teaching objectives, teaching difficulties, teaching method selection, teaching process design, and other links and extracts practical teaching design theory of Ideological and political discipline.

Through the analysis of the monograph on Ideological and political teaching design, the author finds that, in the aspect of ideological and political teaching design in China, we pay attention to practicality. On the basis of studying the theory of teaching design, we attach importance to the connection with the content of Ideological and political teaching and hope to really improve classroom teaching under the guidance of theory. The author has found more than 100 academic papers and periodicals on ideological and political teaching design through CNKI. It can be divided into two major categories: (1) theoretical category. For example, “research on the teaching design of the new ideological and political course” puts forward that cognition and attitude are inseparable in real life and permeate in every activity of people. We can not separate them in thinking just for the completion of teaching tasks. Cognition and attitude are important parts of teaching. Teaching design should pay attention to the integration of the two. “Research on the teaching design of middle school ideological and political course under the new curriculum reform” mentioned that the teaching design should be based on the new curriculum standard, combined with the nature of moral education in ideological and political course, guide teachers' teaching behavior, improve students' bad learning habits, and finally achieve the established teaching goals [8].

(2) For practical operation. Such as Menghongjuan's “how to optimize the teaching design of Ideological and political courses in Colleges and universities,” the teaching design should ensure the effective learning and all-round development of students and design teaching for the active development of students. “Exploration of Ideological and political teaching design in Colleges and universities from the perspective of constructivism” puts forward that teaching design is the presupposition of a class and explains how to clarify the goal analysis, how to guide students' independent exploration, and how to scientifically evaluate students in the process of teaching design. Through the analysis of the relevant literature found in CNKI, the author finds that the research on ideological and political teaching design in China is extremely active, and the relevant design research results are increasing, mainly from front-line teachers, experts, and scholars. They often start from the two aspects of theoretical guidance and practical application, establish a scientific theoretical system of instructional design, and apply the theory to the link of instructional design. At the same time, they also attach importance to the advancement of instructional design and combine modern teaching means to promote teaching optimization [9].

RETRACTED

At present, there are few works on the ideological and political teaching design in colleges and universities under Rogers' humanism, and there are few such papers available. Similar studies that can be used for reference include the following: Xiao Yu paid attention to the relationship between education and teaching and students' all-round development in “the guiding significance of humanistic learning theory to teaching design,” connected with students' personal experience, paid equal attention to cognitive design and emotional design, paid attention to the creation of learning atmosphere and environment, and promoted students' stress free and threat free learning. Shaomingli applied humanism to the teaching design of University Geography in the “teaching design of University Geography from the perspective of humanistic education theory,” guided all links of teaching design through humanistic theory, and tried to realize student-centered classroom teaching: Ma Jinfeng stated in “the Enlightenment of Rogers' Humanistic Learning Theory on education and teaching” that teaching should pay attention to the overall coordinated development of people and cultivate students' creativity and pay attention to the development of potential, and the teaching process and results should reflect the concept of “student-oriented” [10, 11]. In the “teaching design principles based on Humanistic Learning Theory,” Wen Dong proposed student-centered learning, emphasizing personal meaning, creating real problem situations (Figures 5–7), making full use of various learning resources, pursuing the openness of the learning process, advocating collaborative learning, and strengthening the emotional interaction between teachers and students.

To sum up, the existing research on ideological and political teaching design in colleges and universities and the research on teaching design from the humanistic perspective have many research results, which have great reference significance for front-line political teachers to improve their own teaching design. However, there are relatively few researches on ideological and political teaching design based on humanistic theory. Therefore, this paper extracts the essence of Rogers' humanistic theory and specifically infiltrates it into the ideological and political teaching design of colleges and universities, trying to make a breakthrough in this research field [12].

The analysis of the influence of the teaching environment design of College Politics Course under the campus humanistic governance environment needs to be realized by means of multiple linear regression. Assuming conditions, least square estimators, and Gauss Markov theorem to establish a multiple linear regression model, there is the following formula:

(1) $$\begin{array}{c} y_{x}=\beta_{1}x_{a}+\beta_{2}x_{a}+\cdots +\beta_{n}x_{a}+u_{i}. \end{array}$$

In the formula, *y*_*x*_ is the dependent variable, *x*_*a*_ is the independent variable, *u* is the random error term, and *β* is the regression parameter.

RETRACTED

White test is a general heteroscedasticity test (Figure 8). In 1980, it was proposed that the White test did not require any assumptions about the nature of heteroscedasticity but was required to estimate the regression model first.

Based on the linear relationship between the original residual and explanatory variables, the square term and cross term of explanatory variables are added, so the auxiliary regression model is obtained. Testing whether the original model has heteroscedasticity is equivalent to testing whether the regression parameters of the auxiliary regression model are significantly zero except for constants. If *h* holds, it is equivalent to being a constant, and the original model does not have heteroscedasticity; otherwise, the original model has heteroscedasticity [13, 14]. The OLS method is used to estimate the original regression model to obtain the residual square sequence, and then, the auxiliary regression model can be constructed:

(2) $$\begin{array}{c} u_{2}^{i}=f\left(x_{i1},\ldots ,x_{ik},x^{2}{}_{i1},\ldots ,x^{2}{}_{ik},\ldots ,x_{ik-1},\ldots ,x_{ik}\right), \end{array}$$

where *f*(*x*) is a linear function with constant term, and the model is estimated by OLS method to obtain *R*^2^. Given significance level *α*, calculate

(3) $$\begin{array}{c} \text{WT}\left(g\right)={\text{TR}}^{2}. \end{array}$$

Compare it with the critical value *Z* to determine whether to accept the original hypothesis, and then determine whether the original regression model has heteroscedasticity.

Through the previous analysis, we construct the factor model of students' learning politics, which contains the above related explanatory variables. Through the investigation of multiple factors and the dependent variables of students' academic performance, it can be found that there is a multiple linear relationship. The multivariate linear model is established as follows:

(4) $$\begin{array}{c} Y_{i}=\beta_{0}+\beta_{1}x_{1i}+\beta_{2}x_{2i}+\beta_{3}x_{3i}+\cdots +\beta_{n}x_{ni}+u_{i}. \end{array}$$

According to the results output by EViews, the regression standard deviation is obtained *σ*.

(5) $$\begin{array}{c} \text{S.E.of ergression}=8.9349. \end{array}$$

According to the data output by EViews,

(6) $$\begin{array}{c} \text{ESS}=7184.937,\\ \text{R}-\text{squared}=0.6351,\\ \text{Adjusted R}-\text{squared}=0.5986. \end{array}$$

The results show that the estimated regression equation fits the sample data generally. In practical application, generally speaking, the larger the *R* or *R*′ is, the better the model fitting is. However, the size of *R* or *R*^2^ only indicates the goodness of fit of the estimated regression equation to the data of *D* samples under the given sample conditions. We cannot select the model only based on the size of *R* or *R*′. Sometimes, in order to keep the significant explanatory variables in the model, we prefer to sacrifice a little goodness of fit [15, 16].

RETRACTED

## 3. Research Methods

### 3.1. Design of Learning Situation Analysis

Learning situation analysis is an essential part of teaching design, but in the traditional teaching design, learning situation analysis is in a neglected corner. Students should be sincere, receptive, and empathic, which highlights the importance of learning situation analysis in teaching design. Only when teachers understand students' psychology, students' development status, and existing knowledge level can they really see problems from the perspective of students, accept students, create a positive classroom atmosphere with students, and complete learning tasks. The content of ideological and political subject is abstract and general. When designing teaching objectives, teaching methods, and teaching processes, teachers must consider students' acceptance ability and students' development level and reasonably carry out teaching design based on students [17].

### 3.2. Design of Teaching Objectives

Teaching objectives are the purpose of classroom teaching activities, and the basis for determining teaching contents, selecting teaching methods, and evaluating teaching activities. The teaching goal design of Ideological and political course should have the characteristics of comprehensiveness and hierarchy. Comprehensiveness refers to the harmonious unification and overall improvement of knowledge, ability, emotion, attitude, and values. Rogers' theory proposes to cultivate people who act in both cognitive and emotional ways. The realization of this ideal should have a realistic teaching goal. This realistic teaching goal not only can rely on the past knowledge goal, but also needs the ability goal and the emotional attitude value goal [18]. See Figure 9 for the design process of teaching objectives.

Goals are not separate; they need to be interconnected and integrated. In the design of ideological and political teaching objectives, teachers need to consider what the teaching knowledge points are and what the key contents are. Next, they need to think about which teaching materials to choose to connect with the teaching content. At the same time, such teaching can cultivate students' abilities and develop their emotions. Hierarchy means that the design of teaching objectives reflects individual differences and teaches students according to their aptitude. Each student has differences in personality, ability, cognitive style, etc., which means that, under the class teaching system, students can not complete the same learning tasks, and the gap between students will be widened in the collective class with the same goal. Rogers' theory advocates taking students as the center. He hopes that every student can find a sense of achievement in the classroom, which requires that the teaching objectives have levels and can meet the needs of students with different ability levels. When designing the ideological and political teaching objectives, we should analyze the teaching contents in detail and refine the teaching objectives at different levels, from low-level to high-level. Each student has a learning task that can be pursued and can reach their own recent development zone [19, 20].

RETRACTED

### 3.3. Design of Teaching Methods

Teaching method is a common activity way for teachers and students to complete teaching tasks. So, the design of teaching method should be carried out from two angles, that is, the method of teachers' teaching and the method of students' learning. Rogers' theory puts forward “nondirective teaching,” which requires enlightening teaching methods and uses various means to mobilize students' initiative and enthusiasm in learning. The method of learning should encourage students to actively participate in the classroom, excavate the connotation of knowledge, and complete the learning task through independent, cooperative, and exchange learning methods. For ideological and political teaching design, teachers should formulate students' study plans according to curriculum standards, teaching materials, and learning conditions. The study plans should involve situational enlightenment, reading carding, and ability testing and be connected through questions. According to the problems in the study plan, students can consult textbooks, find materials, and complete preliminary learning tasks. For places they do not understand, they should mark them to improve their independent learning ability. More importantly, they should stimulate their curiosity and thirst for knowledge about problems they do not understand. For the problems in the process of self-study, teachers divide learning groups, and the groups share resources and help each other to solve their puzzles in the learning plan. For the problems that are difficult to solve, the teacher creates a situation and organizes exploration and solution.

RETRACTED

### 3.4. Design of Teaching Content

Ideological and political teaching content is the basis of political classroom activities and the task that students need to complete in their learning activities. It comes from textbooks, but it is higher than textbooks. It answers the questions of what teachers teach and what students learn. Rogers' humanism advocates cultivating “complete people.” Students get all-round development in the process of learning, and they can adapt to the society even out of the classroom. Therefore, teachers should pay attention to selecting teaching materials from life to reflect the authenticity, so that students can feel the charm of knowledge in the real situation, use knowledge to solve practical problems, and develop their ability.  Figure 10 shows common teaching methods.

At the same time, we should also pay attention to the impact of the teaching content on students' emotions, attitudes, and values, make use of the characteristics of the political discipline, cultivate students' due political ideology, political culture, and political consciousness, and improve students' humanistic feelings. Regarding the choice of ideological and political teaching content, teachers need to go into life, from the political, economic, and cultural aspects, to collect teaching materials, select some cases with educational significance and combine them with teaching, recombine the teaching contents, combine the difficult contents in the teaching objectives with cases, create life scenes, and help students understand.

### 3.5. Teaching Process Design

Teaching process design is the key part of teaching design. It is a design process for teachers to design teaching tasks according to their own educational ideas and classroom teaching objectives. It is a detailed description of teaching links. Teachers' teaching ideas are embodied in the design of teaching process. The main task of traditional teaching process design is to require students to master the test site. Students are regarded as the storage box of knowledge, ignoring students' participation and emotional needs. In the teaching process under Rogers' theory, the teacher is a guide, and the students are the main body of the classroom. Teachers should pay attention to every student, establish a multidirectional communication mode between teachers and students, treat students equally, encourage students to express their real ideas, and develop them in the communication and interaction.  Figure 11 shows the common teaching process.

The design of ideological and political teaching process should highlight two points: one is student participation, and the other is link design. Students are the main body of learning activities. Only with the participation of students can learning activities really have a soul. In the design of teaching process, there should be a process of students' autonomy, cooperation, and exploration, so that students can have the opportunity to express their ideas. At the same time, in view of the abstract and general characteristics of ideological and political learning content, only students' positive thinking can truly grasp knowledge and develop emotion. Link design is a feature of the design of Ideological and political teaching process. The ideological and political learning content has an internal logic system, which requires teachers to grasp the teaching process as a whole, consider the students' cognitive characteristics, pay attention to the fluency between links, make links, attract students' attention, and help students understand.

RETRACTED

### 3.6. Design of Teaching Evaluation

The teaching evaluation involved in this subject is mainly aimed at the evaluation of students' learning activities and learning effects in teaching design. It is an indispensable feedback link in the learning process. The fundamental purpose of teaching evaluation is to promote students' development. The process evaluation of teaching should gradually replace the summary evaluation.  Figure 12 shows the teaching effect evaluation model:

If there are problems beyond the learning content in the teaching process, teachers' educational wit should be brought into play to give evaluation and guidance, instead of turning a blind eye to them. For the evaluation of students, we should advocate the diversification of evaluation subjects, teachers' evaluation is the foundation, students' mutual evaluation is the auxiliary, students' self-evaluation is the fundamental, and we give full play to the role of collective education and self-education. Teaching evaluation should also pay attention to individual differences and combine students' own reality to teach students in accordance with their aptitude. Ideological and political education also has a unique moral nature. Therefore, teaching evaluation has a directionality. It should not only focus on the results, but also pay attention to the ideological guidance, so as to achieve the combination of knowing and doing imperceptibly.

## 4. Result Analysis

The 10-point system is used to score the impact of teaching environment design. 0 is the lowest, representing the most dissatisfied, and 10 is the highest, representing the most satisfied. The specific scores are calculated by SPSS 21.0 and expressed in mean ± standard deviation. The results are as follows:

RETRACTED

### 4.1. The Impact of Teaching Environment Design on the Satisfaction Score of Teaching Methods and Means

After the design of the teaching environment, the teachers' scores for the vivid and intuitive teaching methods and means, method innovation, teacher-student interaction, and knowledge development are (8.21 ± 1.22), (7.84 ± 1.20), (9.25 ± 0.12), and (9.10 ± 0.51), respectively. Students' scores were (8.65 ± 4.10), (8.52 ± 1.00), (9.33 ± 0.16), and (8.77 ± 0.54), respectively. See Table 1.

### 4.2. Impact of Teaching Environment Design on Teaching

After the design of the teaching environment, the teachers' scores for Mandarin teaching, proper behavior, clear concept, and adequate preparation are (9.14 ± 0.41), (8.74 ± 1.33), (9.00 ± 0.33), and (9.47 ± 0.69), respectively. Students' scores were (9.51 ± 0.28), (8.74 ± 1.25), (9.46 ± 0.20), and (8.68 ± 0.25), respectively. See Table 2.

### 4.3. Influence of Teaching Environment Design on Teaching Attitude

After the design of the teaching environment, the teachers' scores for serious attitude, clear purpose, good self-cultivation, and good discipline are (9.80 ± 0.20), (9.00 ± 0.12), (8.69 ± 0.74), and (8.99 ± 0.25), respectively. Students' scores were (9.54 ± 0.10), (9.00 ± 0.87), (9.62 ± 0.11), and (8.74 ± 0.65), respectively. See Table 3.

### 4.4. Impact of Teaching Environment Design on Teaching Management

After the design of the teaching environment, the teachers' scores are (7.49 ± 2.00) and (9.23 ± 0.15) for the strict and patient requirements of teaching management. The students' scores were (8.74 ± 0.62) and (9.33 ± 0.21), respectively. See Table 4.

### 4.5. Impact of Teaching Environment Design on Teaching Quality

After the design of teaching environment, among the scores of good academic performances, enhanced students' ability, more learning gains, and improved students' interest in teaching quality, teachers' scores are (8.59 ± 0.80), (9.16 ± 0.17), (8.43 ± 0.36), and (8.29 ± 0.89), respectively. Students' scores were (9.10 ± 0.33), (9.28 ± 0.44), (9.16 ± 0.27), and (8.35 ± 1.20), respectively. See Table 5.

## 5. Conclusion

The new curriculum reform puts forward the slogan of “for the rejuvenation of the Chinese nation, for the development of each student” for the cultivation of students. The teaching design based on Rogers' humanistic theory is the embodiment of this idea. It respects the dominant position of students, pays attention to the integration of knowledge and practice of students, develops students' potential in the learning process, and sublimates students' emotions in the learning process. Teaching design is the teacher's advance planning for classroom teaching and the embodiment of professional quality. An excellent teacher should have his own style of teaching mathematics and his own characteristics of teaching design. This paper summarizes the main points from Rogers' humanistic theory, analyzes some problems in the current ideological and political teaching design in colleges and universities according to the main points, and puts forward the principles of teaching design. This paper puts forward new ideas from the perspectives of learning situation design, goal design, method design, content design, process design, and evaluation design, so that teachers can truly achieve “student-oriented” in teaching design and truly realize the comprehensive and harmonious development of students' knowledge goals, ability goals, emotional attitudes, and values.

RETRACTED

## Figures and Tables

**Figure 1:** Teaching design process.

**Figure 2:** Humanistic theory.

**Figure 3:** Cognitive theory.

**Figure 4:** College students' thinking on e-learning.

**Figure 5:** Proportion of situational teaching method in each teaching link.

**Figure 6:** Presentation of situational teaching method.

**Figure 7:** Life atmosphere of situational teaching method.

**Figure 8:** Schematic diagram of regression model.

**Figure 9:** Design process of teaching objectives.

**Figure 10:** Common teaching methods.

**Figure 11:** Common teaching process.

**Figure 12:** Teaching effect evaluation model.

**Table 1:** Influence of teaching environment design on the score of satisfaction with teaching methods and means.

Teaching methods and means	Teacher rating	Student rating
Vivid and intuitive	8.21 ± 1.22	8.65 ± 4.10
Method innovation	7.84 ± 1.20	8.52 ± 1.00
Teacher student interaction	9.25 ± 0.12	9.33 ± 0.16
Knowledge development	9.10 ± 0.51	8.77 ± 0.54

**Table 2:** Influence of teaching environment design on Teaching.

Teaching situation	Teacher rating	Student rating
Putonghua teaching	9.14 ± 0.41	9.51 ± 0.28
Good manners	8.74 ± 1.33	8.74 ± 1.25
Clear concept	9.00 ± 0.33	9.46 ± 0.20
Well prepared	9.47 ± 0.69	8.68 ± 0.25

**Table 3:** Influence of teaching environment design on teaching attitude.

Teaching attitude	Teacher rating	Student rating
Serious attitude	9.80 ± 0.20	9.54 ± 0.10
Definite purpose	9.00 ± 0.12	9.00 ± 0.87
Well cultivated	8.69 ± 0.74	9.62 ± 0.11
Good discipline	8.99 ± 0.25	8.74 ± 0.65

**Table 4:** Influence of teaching environment design on teaching management.

Teaching management	Teacher rating	Student rating
Strict requirements	7.49 ± 2.00	8.74 ± 0.62
Patience	9.23 ± 0.15	9.33 ± 0.21

**Table 5:** Influence of teaching environment design on teaching quality.

Teaching quality	Teacher rating	Student rating
Good academic performance	8.59 ± 0.80	9.10 ± 0.33
Students' ability enhancement	9.16 ± 0.17	9.28 ± 0.44
Learn more	8.43 ± 0.36	9.16 ± 0.27
Improvement of students' interest	8.29 ± 0.89	8.35 ± 1.20

RETRACTED

## Data Availability

The labeled data set used to support the findings of this study is available from the corresponding author upon request.
